The article "Cytotoxicity Analysis of Three Bacillus thuringiensis Subsp. israelensis δ-Endotoxins towards Insect and Mammalian Cells" was published in 2012. Journal: PLoS One.

# Cytotoxicity Analysis of Three *Bacillus thuringiensis* Subsp. *israelensis* δ-Endotoxins towards Insect and Mammalian Cells

**DOI:** 10.1371/journal.pone.0046121

**Published:** 2012-09-21

**Authors:** Roberto Franco Teixeira Corrêa, Daniel Mendes Pereira Ardisson-Araújo, Rose Gomes Monnerat, Bergmann Morais Ribeiro

**Affiliations:** 1 Departamento de Biologia Celular, Universidade de Brasília, Brasília, Distrito Federal, Brazil; 2 Embrapa – Recursos Genéticos e Biotecnologia, C.P. 02373, Brasília, Distrito Federal, Brazil; Universidad Nacional Autonoma de Mexico, Instituto de Biotecnologia, Mexico

## Abstract

Three members of the δ-endotoxin group of toxins expressed by *Bacillus thuringiensis* subsp. *israelensis*, Cyt2Ba, Cry4Aa and Cry11A, were individually expressed in recombinant acrystalliferous *B. thuringiensis* strains for *in vitro* evaluation of their toxic activities against insect and mammalian cell lines. Both Cry4Aa and Cry11A toxins, activated with either trypsin or *Spodoptera frugiperda* gastric juice (GJ), resulted in different cleavage patterns for the activated toxins as seen by SDS-PAGE. The GJ-processed proteins were not cytotoxic to insect cell cultures. On the other hand, the combination of the trypsin-activated Cry4Aa and Cry11A toxins yielded the highest levels of cytotoxicity to all insect cells tested. The combination of activated Cyt2Ba and Cry11A also showed higher toxic activity than that of toxins activated individually. When activated Cry4Aa, Cry11A and Cyt2Ba were used simultaneously in the same assay a decrease in toxic activity was observed in all insect cells tested. No toxic effect was observed for the trypsin-activated Cry toxins in mammalian cells, but activated Cyt2Ba was toxic to human breast cancer cells (MCF-7) when tested at 20 µg/mL.

## Introduction

Crop-damaging insects are responsible for a significant decrease in world crop yields every year [1]. Insects are also important vectors of human disease and thus are the focus of considerable control efforts [2]. The use of biological control of insects has been shown to be a safe, successful, cost-effective and promising alternative to chemical control [3]. The gram-positive, spore-forming bacterium *Bacillus thuringiensis* (Bt), which occurs naturally in several environments [4], is largely employed in biological control of various insect pests. Different Bt subspecies are toxic to specific insect groups, producing, during the sporulation phase, crystalline inclusion bodies consisting of host-specific insecticidal Cry and/or Cyt proteins known as δ-endotoxins [5]. Due to the high specificity to target insects and little evidence of toxicity to vertebrates and plants, the use of Bt as an alternative to chemical insect control has increased greatly [6]. Cry protoxins are solubilized under alkaline pH in the insect midgut and activated by endogenous gut proteases; these protoxins then interact with specific receptors present in the epithelial cells of the insect midgut, causing pore formation and consequent osmotic cell lysis [7], [5]. Cyt protoxins also need solubilization and proteolytic cleavage in the insect’s midgut to become active, but in contrast to Cry toxins, Cyt proteins bind nonspecifically to unsaturated phospholipids present in the host’s epithelial cell, forming pores [8] or disrupting the membrane through a detergent-like mode of action [9]. Relevant differences in the midgut physiology and consequent variation in proteolytic activity among different insect orders may determine the specificity of each toxin. For example, the main digestive lepidopteran and dipteran proteases are serine-proteases, whereas those found in coleoptera are cysteine and aspartic-proteases [10]. Cyt proteins are toxic to mosquito larvae, although their toxicities are usually lower than those from Cry proteins toxic to dipteran larvae [11]. It has also been reported that native toxins belonging to the Cyt family are toxic *in vitro* to erythrocytes and other mammalian cells, and lethal to mice after intravenous injection [12]–[15]. Cyt toxins have been shown to act synergistically with mosquitocidal Cry toxins [16]; Cyt1Aa can, for example, function as a receptor for the binding of Cry11Aa to *Aedes aegypti* gut cell membranes [17], thus playing a crucial role in the general activity of the parasporal inclusion. *Bacillus thuringiensis* subsp. *israelensis* (Bti) is highly toxic to dipteran insects and is utilized in mosquito control in many countries [18] e.g., to combat malaria and dengue fever. The entomopathogenic activity of Bti for *Culex spp*, *Aedes spp* and *Anopheles spp* is due to the presence of a megaplasmid, pBtoxis, which encodes at least four Cry and two Cyt toxins: Cry4Aa, Cry4Ba, Cry10, Cry11Aa, Cyt1Aa and Cyt2Ba [19]. This plasmid also contains coding sequences for two other proteins (P19 and P20) believed to act as chaperones, helping toxin crystal formation [19].

In our study acrystalliferous Bt strains were engineered to individually express Cry4Aa, Cry11A and Cyt2Ba proteins; the strains could then be tested *in vitro* against different cultured cell lines to determine their individual toxic activity and possible synergistic interactions with other toxins under controlled experimental conditions.

## Results and Discussion

### Bti Toxin Genes

Blast analysis of the sequences from amplified Bti genes showed that the *cyt2Ba* gene was identical to the sequence described elsewhere [20] (Genbank accession number = U52043), except for a 6xHis tag sequence in the N-terminal end, introduced by a PCR primer. The *cry11A* gene showed 100% nucleotide sequence identity with the *cry11A* gene described earlier by Berry *et al.* [19] (Genbank accession number = AL731825). The *cry4Aa* gene showed 98% nucleotide sequence identity with the first described *cry4Aa* gene [21] (Genbank accession number = Y00423) with eight nucleotide base differences, resulting in eight amino acid changes at the following positions: S16T, E32G, T301P, F569L, H572R, D980N, F1168V, I1170K.

### Expression, Purification and Solubilization of Cyt and Cry Toxins

The amplified DNA fragments containing the *cyt2BaHis*, *cry11A* and *cry4Aa* coding sequences were first cloned in a PCR cloning vector (not shown), then transferred to the binary *B. thuringiensis* expression vector pSVP27A under control of the sporulation phase promoter *Pcyt* (Figures 1A, B, and C). The recombinant plasmids were purified and inserted into an acrystalliferous Bt by electroporation, giving rise to the recombinant BtCyt2BaHis, BtCry11A and BtCry4Aa strains. The recombinant colonies were grown in selective media for 72 h and the spore/crystal of the mixture was subjected to centrifugation in discontinuous sucrose gradients.

**Figure 1:** Schematic linear representation of the expression plasmids and SDS-PAGE analysis of Cry11A, Cry4Aa and Cyt2Ba expression. Panels A, B and C: *cyt2BaHis*, *cry4Aa* and *cry11A* genes inserted, respectively, into the *Bam*HI cloning site of the pSVP27A plasmid. The recombinant genes are under the control of a sporulation phase promoter, Pcyt. The genes for positive clone selection in *E. coli* (Amp-r) and in *B. thuringiensis* (CAT-r) are shown. Selected restriction enzyme sites used to confirm cloning are also shown. Panels D and E: SDS-PAGE of purified protoxins (Cry11A, Cry4Aa and Cyt2Ba) from recombinant *B. thuringiensis* strains. As a control, a sporulated acrystaliferous *B. thuringiensis* strain (4Q7) extract was used. Selected molecular masses of the protein markers are shown (ColorPlus™ Prestained Marker-NEB, panel D and BenchMark™ Protein Ladder-Invitrogen, Panel E) on the left side of both panels.

After purification, Cry11A and Cry4Aa crystals were solubilized and analyzed by SDS-PAGE. Protein bands with the expected molecular masses were detected (66 kDa and 130 kDa, respectively) (Figure 1D). Despite the absence of the accessory proteins P20 and P19, usually associated with the folding of Cry11A, the recombinant Cry11A protein was largely expressed with the expected molecular mass. Xu *et al.* [22] have shown that the Cry11A protein was successfully expressed in recombinant *E. coli,* in the presence or absence of P20. On the other hand, in another recombinant Gram-negative bacterium, *Pseudomonas putida*, the Cry11A protein was produced in satisfactory amounts only when P20 was co-expressed [22]. Furthermore, high levels of Cry11A expression and toxic activity against *A. aegypti* larvae were shown in a recombinant acrystalliferous Bt strain, 4Q2-81 [18]. In our work the Cyt2BaHis protein was obtained by centrifugation of the recombinant Bt extracts in a discontinuous sucrose gradient, followed by solubilization with Na_2_CO_3_ and affinity chromatography due to the large number of contaminants present after centrifugation (data not shown). After this additional purification step, SDS-PAGE analysis was carried out, showing a single 27 kDa band as expected (Figure 1E).

**Figure 2:** Cytotoxicity assays in insect cell cultures and western blot analysis of Cyt2Ba activation. Panel A: 20 µg/mL of each activated toxin, Cry4Aa and Cry11A, were incubated with different insect cell lines for 30 min. Untreated cells (control) were not incubated with any of the toxins. The percentage of cytotoxicity (cell mortality) was determined by luminometric readings based on luciferase activity. Panel B: Trypsin activation of Cyt2BaHis was proceeded and both protoxin and the activated toxin samples were analyzed by western blot with an anti-His antibody. The arrow shows a band of 27 kDa expected for the non-activated protein. The proteolytic cleavage of Cyt2BaHis resulted in the 6xHis tag loss, making the activated toxin undetectable in western blot analysis using anti-His antibody. Panel C: The activated Cyt2Ba toxin was incubated with insect cells at two different concentrations (5 and 20 µg/mL). Cytotoxicity was determined as for panel A. Panel D: Combinations of Cyt2Ba (5 µg/mL) and the two Cry toxins (20 µg/mL for each toxin) were incubated with insect cell lines. Cytotoxicity percentages were measured according to the same method employed in panel A and C. The toxins concentrations are shown in brackets. One type of dipteran cells (C6/36) and three types of lepidopteran cells (Ld, Sf-21 and Bm) are shown on the cytotoxicity assays graphics.

### Toxicity of Dipteran-specific Cry4Aa and Cry11A Proteins to Dipteran and Lepidopteran Cell Lines

Cry4Aa and Cry11A proteins have been shown to be toxic to mosquitoes *in vivo* [4], [23], [24], [25]. Our study used these two δ-endotoxins in cytotoxicity assays against both lepidopteran and dipteran cell cultures. Solubilized and trypsin-activated Cry4Aa and Cry11A toxins were incubated, separately or in combination, with dipteran and lepidopteran cells. Use of equal amounts of Cry4Aa and Cry11A toxin (20 µg/mL) resulted in similar toxic effects in all cells tested. A slightly significant difference in toxicity was observed only when the toxins were tested separately against lepidopteran IPLB-SF-21AE and IPLB-LD-652Y cells. Interestingly, the mixture of the two toxins showed higher toxic activity to all insect cell lines (Figure 2A). In contrast, Chilcott and Ellar [26] observed no cytotoxicity when incubating trypsin-activated 130 kDa and 65 kDa Bti proteins with a cell line derived from *A. albopictus*. In our assays, the Cry4Aa and Cry11A activated toxins showed 10 to 15% of the toxicity of wild type Bti-activated toxins (see below) in *A. albopictus* C6/36 cells. Furthermore, the mixture of the two recombinant proteins increased toxicity to approximately 36% of the wild type Bti-activated toxins. As reported earlier [27], different cell lines from *Choristoneura fumiferana* (spruce budworm) showed distinct relative susceptibility when incubated with Bt activated δ-endotoxins. The presence, absence or availability of suitable receptors on the cell surface could explain the diverse levels of susceptibility among different cell lines deriving from one insect species. The increased toxicity of combined Cry4Aa and Cry11A to *A. albopictus* cells was also observed in previous research [18]. The earlier study showed lower individual toxicity for Cry4Ba, Cry4Aa and Cry11Aa proteins to fourth-instar *A*. *aegypti* than native crystals produced by Bti. Sauka *et al*. [28] demonstrated that a mixture of Cry1Ba and Cry1Da toxins yielded a synergism factor higher than 1 [29] when tested against neonate larvae of *Epinotia aporema* (bean shoot borer), suggesting a possible synergism between these Cry toxins. However, no synergistic interaction between 130kDa and 65 kDa Cry proteins was detected *in vivo* against *A. aegypti* larvae [26], [29]. Although Cry4Aa and Cry11A protoxins used in our work may share the same molecular mass as the respective proteins reported previously by other research groups, they are not the same polypeptides; there may be differences in the specificity of the molecular interactions. Using a model for synergism proposed by Tabashnik [29], we calculated the synergism factor (SF) for the Cry4Aa and Cry11A mixture in all cell lines tested. For this purpose, the median lethal concentration (LC_50_) was estimated (Table 1). For the dipteran C6/36 and the lepidopteran SF-21 cell lines, the SF was higher than 1, suggesting possible synergistic effects (Table 2). Poncet *et al*. [30] detected higher SF values, and thus, stronger synergism when using a mixture consisting of Cry4A and Cry11A against three different species of mosquito larvae. The dipteran cell line used in our assays, *in vitro*, is not necessarily derived from the midgut, but from a minced *A. albopictus* larvae. In contrast, the SF was lower than 1 for the mixture with the other two lepidopteran cell lines tested (Ld and Bm5) and some antagonism was detected (Table 2). Purified crystals from wild type Bti, containing all the δ-endotoxins expressed by this bacterium, were solubilized and added separately to the cell cultures at a concentration of 5 µg/mL. This amount of solubilized protein caused 100% cell lysis (data not shown) and was used as a positive reference in the cytotoxicity studies.

**Table 1:** Cytotoxicity of mixtures of Cry and Cyt toxins of *Bacillus thuringiensis* subsp. *israelensis* to insect cell lines.

	Cry4Aa/Cry11A			Cyt2Ba/Cry11A			Cyt2Ba/Cry4Aa		
	LC_50_ a (95% limits)	S.^b^	X^2c^	LC_50_ a (95% limits)	S.^b^	X^2c^	LC_50_ a (95% limits)	S.^b^	X^2c^
C6/36	59.46 (49.48–80.261)	2.07	0.77	61.44 (53.27–74.65)	2.44	2.30	78.96 (66.60–105.51)	2.52	2.17
Bm5	111.65 (99.23–132.47)	3.29	1.34	147.03 (93.77–618.44)	1.45	0.68	59.93 (46.96–92.23)	2.47	3.31
Ld	108.97 (78.45–274.18)	2.07	4.40	54.79 (43.11–78.29)	2.50	3.62	106.47 (79.75–200.03)	1.81	1.30
Sf	75. 85 (50.66–119.51)	2.20	4.30	55.47 (44.41–76.275)	2.63	3.31	97.45 (73.02–175.76)	1.68	1.76

a -mean lethal concentration. Numbers in parentheses are 95% fiducial limits.

b -slope.

c -chi-square.

**Table 2:** Observed and expected cytotoxicity of Cry and Cyt toxin mixtures to insect cell lines and the calculated synergism factor.

	Cry4Aa/Cry11A			Cyt2Ba/Cry11A				Cyt2Ba/Cry4Aa			
	LC_50_ a	Exp. LC_50_ b	SF^c^		LC_50_ a	Exp. LC_50_ b	SF^c^	LC_50_ a	Exp. LC_50_ b	SF^c^	
C6/36	59.46	77.70	1.30		61.44	74.92	1.21	78.96	81.54	1.03	
Bm5	111.65	100.7	0.89		147.03	95.67	0.65	59.93	91.94	1.53	
Ld	108.97	65.47	0.60		54.79	55.45	1.01	106.47	89.64	0.84	
Sf	75. 85	75.85	1.10		55.47	76.45	1.37	97.45	97.48	1.01	

a -observed mean lethal concentration (µg/mL).

b -expected mean lethal concentration (µg/mL).

c -synergism factor.

### Cyt2Ba Cytotoxicity to Insect Cells

Although Cyt toxins are produced by some dipteran-specific Bt strains [31], [32], these toxins have been reported to be cytolytic to a broad range of cells [12]. To determine any possible relationship between dose and toxicity to different cell lines, we activated purified Cyt2Ba toxin (Figure 2B), which has been proposed to bind cell membranes in a non-specific manner [8], and incubated it with four types of insect cells using two different concentrations (5 or 20 µg/mL). As demonstrated in our assays, Cyt2Ba showed toxicity to all insect cells tested (Figure 2C). There was also a significant increase in the toxic activity when Cyt2Ba was used at a concentration of 20 µg/mL.

### Incubation of Cell Lines with Both Cry and Cyt Toxins

To verify that Cyt2Ba and Cry toxins (Cry4A and Cry11A) interact cytotoxically, assays were performed using combinations of these toxins. The Cry toxins were used at a concentration of 20 µg/mL, whereas the Cyt2Ba toxin was used at 5 µg/mL, since any increase in the obtained cytotoxicity could be misinterpreted as activity of only Cyt2Ba at its highest concentration (Figure 2C).The data showed a higher level of toxic activity when Cry11A and Cyt2Ba were used in combination (Figure 2D). In all cells tested the toxicity demonstrated by this combination was significantly higher than the Cry4Aa and Cyt2Ba combination (Figure 2D). Nevertheless, in both cases different types of toxic interactions were observed when determining the LC_50_ of the mixtures and calculation of SF values (Tables 1 and 2). SF >1 was achieved with the mixture Cyt2Ba/Cry11A in dipteran C6/36 and lepidopteran Sf-21 cells as well as with the mixture Cyt2Ba/Cry4Aa in lepidopteran Bm5 cells. These data indicate synergism between the Cyt and Cry toxins tested, which agrees with other works showing this kind of interaction [33], [16]. Weak additive effects (SF ∼ 1) were obtained for the Cyt2Ba/Cry11A mixture when it was tested against lepidopteran Ld cells. Similar SF values were detected after incubation of Cyt2Ba/Cry4Aa with C6/36 and Sf-21 cells. It was also demonstrated that some antagonism (SF lower than 1) may occur between Cyt and Cry toxins depending on the cell line tested. SF <1 was observed for the Cyt2Ba/Cry11A mixture in Bm5 cells and for Cyt2Ba/Cry4Aa in Ld cells. Hughes *et al*. [34] also showed slight antagonism *in vivo* when Cry11A and Cry4B were assayed in combination with Cyt1A against *Chironomus tepperi* (Diptera: Chironomidae). Aside from this report, it has been demonstrated that binding of Cry11Aa to *A*. *aegypti* membranes is greatly enhanced by preincubation of “brush border membrane vesicles” (BBMVs) with Cyt1A [17]. Except for the C6/36 cells, our combination of the three toxins (Cyt2Ba, Cry4Aa and Cry11A) led to a decrease of the toxic activity in relation to the Cry11A and Cyt2Ba mixture (Figure 2D). These results indicate that Cyt2Ba acts as a receptor for both Cry toxins, as shown by Pérez *et al*. [17], and Cry4Aa competes with Cry11A for the binding to Cyt2Ba, leading to a weaker interaction than that of Cyt2Ba and Cry11A. There is also evidence that Cry toxins may interact, forming hetero-oligomers *in vivo* [35]. In our work, such molecular interactions between Cry toxins could be more or less effective depending on the cell line tested, after the putative binding of Cry toxins to Cyt2Ba. This may explain why the cytotoxicity of the three toxins together did not decrease in C6/36 in contrast to the other insect cell lines.

### Cry4Aa and Cry11A Toxic Activity When Processed by Lepidopteran Gastric Juice

The Cry4Aa and Cry11A protoxins were also processed by proteases found in the gastric juice extracted from *S. frugiperda* larvae. As previously described, besides the three-domain based structure and the intrinsic amino acid sequence, proteolytic activation is a relevant factor for the toxicity of Cry toxins [36], [37]. The same incubation conditions as well as the protein ratio used for trypsin activation were maintained for gastric juice (GJ) protein processing. The cleavage pattern obtained for Cry4Aa and Cry11A after incubation with *S. frugiperda* midgut proteases resulted in a different SDS-PAGE banding profile than with trypsin activation (Figure 3). According to Christeller *et al.* [38], the GJ from different lepidopteran larvae contain predominantly alkaline proteases with different patterns of trypsin- or chymotrypsin-like activities. Although both types of proteases are members of the serine protease group, Cry proteins may undergo different proteolytic processing upon trypsin or chymotrypsin treatment. For instance, Cry3Aa toxin produced different polypeptides after treatment with each protease, but retained its ability to bind Colorado potato beetle’s (*Leptinotarsa decemlineata*) BBMVs. In contrast, the Cry3Ba toxin was unable to bind *L. decemlineata*’*s* BBMVs using identical proteolytic treatments [39]. In our work, the processed toxins were dialyzed and incubated with insect cell cultures at a concentration of 20 µg/mL. To ensure that neither trypsin nor GJ was responsible for any toxic activity to the cells, cytotoxicity was measured after incubation of both proteases with the cell lines. No cytotoxicity was detected for the processed Cry toxins or for the protease samples (data not shown). Furthermore, Cry11A and Cry4Aa crystals and GJ-activated proteins (20 µg/mL) were also tested *in vivo* against second-instar larvae of *A. aegypti*. Cry11A and Cry4Aa were toxic to *A. aegypti* larvae with LC_50_ values of 53.72 ng/mL and 92.24 ng/mL, respectively (Table 3). In contrast, no toxic activity was observed for the one-dose bioassay using GJ- activated proteins (data not shown). It is possible that the new cleavage pattern yielded by the lepidopteran gastric juice does not provide a functional structure of an active toxin [25]. However, we cannot rule out the possibility that Cry proteins were overdigested by insect gastric juice and consequently inactivated the toxins.

**Figure 3:** SDS-PAGE analysis of Cry4Aa and Cry11A proteolytic activation. The solubilized Cry4Aa and Cry11A protoxins were activated either by standard incubation using trypsin (T) or by using *S. frugiperda’* gastric juice (GJ). The processed proteins were stained with Coomassie blue. Molecular masses in kDa are shown on the left (Prestained Protein Molecular Weight Marker, Fermentas).

**Table 3:** Toxicity of individual Cry proteins to second-instar larvae of *A.aegypti.*

Toxin	n*	LC_50_ (95% limits)**	σ***
Cry11A	75	53.72 (25.13–86.54)	3.814
Cry4Aa	75	92.24 (55.64–123.58)	2.673

* : number of tested larvae;

** : mean lethal concentration for 50% of larvae exposed (µg/mL).

*** σ: standard deviation.

### Cytotoxic Activity of Cry4Aa, Cry11A and Cyt2Ba to a Mammalian Cell Line

The specificity of Cry proteins is also due to the fact that, when ingested by susceptible insect larvae, each toxin binds to specific receptors on the midgut epithelial cell brush border membrane [40]. Thomas and Ellar showed that the pool of purified and solubilized crystal proteins of Bti was toxic to mouse fibroblasts, primary pig lymphocytes and mouse epithelial carcinoma cell lines [12]. To determine whether the dipteran-specific toxins, Cry4Aa and Cry11A, are toxic to mammalian cells via trypsin activation, we performed cytotoxicity assays with human breast cancer cells, MCF-7 (Figure 4). Some Bt strains have been reported to produce parasporal proteins that are capable of discriminately killing cancer cells [41], [42]. However, this anticancer activity is achieved by a different category of parasporal proteins, the so-called parasporins, which exhibit very low homologies (<25%) to Cry and Cyt proteins [42], [43]. Since the wild type Bti δ-endotoxins used here as our positive reference control did not yield 100% mortality when observed by light microscopy, a lysis buffer was added to the cell culture so that all cells were lysed and a reliable reference value was obtained by luminometric reading. No cytotoxicity was detected when any of the Cry4Aa and Cry11A-activated toxins were incubated individually or in combination with the human cells. Mammalian cells do not display receptors for the binding of Cry toxins on their surfaces, which may explain why Bt is not toxic to mammals. In addition, the Cyt2Ba toxin was incubated at two different concentrations with MCF-7 cells (Figure 4). This experiment demonstrated that Cyt2Ba was cytotoxic only at the highest concentration used in our assays (20 µg/mL). This toxicity is probably due to the ability of Cyt2Ba to bind cell membranes without specific receptors. The activity value shown for the activated toxins expressed by Bti, approximately 70% (Figure 4), may be explained by the synergistic effects among additional toxins in the Bti crystals [11]. (For instance, Cyt1Aa has been shown to synergize Cry4 and Cry11 toxins in *A. aegypti* gut cells [17].) To investigate this hypothesis, another cytotoxic assay was carried out using 20 µg/m concentrations of the three toxins (Figure 4) in combination. The mixture of Cry and Cyt toxins showed higher toxicity to MCF-7 cells than Cyt2Ba alone, but non-parametric variance analysis of the cytotoxicity values demonstrated that there was no significant difference in toxicity between Cyt2Ba alone and in combination with the two Cry toxins. It is not clear whether the significantly higher cytotoxic value obtained for a 60 min incubation period was due to the combination of the three toxins. Despite the variance, the cytotoxic effect measurements plotted in the graph (Figure 4) suggest an interaction between the Cry toxins with Cyt2Ba. If this is true, Cyt2Ba may be functioning as a receptor for Cry4Aa and Cry11A, which could lead to pore formation in human cell membranes. Further work is needed to characterize the toxicity interactions between Cry and Cyt proteins in mammalian cells.

**Figure 4:** *In vitro* analysis of Cry and Cyt toxicity to MCF-7 human cells. The percentage of cytotoxicity (cell mortality) was obtained by luminometry for all assays. Individual trypsin-activated Cry4Aa or Cry11A as well as the mixture of these two toxins were incubated with MCF-7 cell cultures for 30 min. Cyt2Ba and isolated crystals of Bti were activated by trypsin and assayed against MCF-7 cells for 30 min. Combinations of the three trypsin activated toxins (Cry4Aa, Cry11A and Cyt2Ba) were incubated with MCF-7 cells for two distinct periods of time (30 and 60 min) and cytotoxicity was measured to verify any variation of toxic activity related to time of incubation. Untreated cells (control) were not incubated with any of the toxins. Concentrations of toxins are in parentheses.

### Conclusion

During evolution insects from different orders and species developed differences in the enzymatic composition of gastric juices in order to adapt to a wide variety of diets. Microorganisms with entomopathogenic capabilities, such as Bt, may have co-evolved to take advantage of digestive enzymes evolved in insect midguts. The toxicity of Bt to insects is chiefly based on δ-endotoxins that must be processed correctly in the intestinal lumen of susceptible insects. The specificity of Cry toxins is, in part, due to the type of proteolytic cleavage that takes place in the insect midgut, as well as to the presence of specific receptors on the midgut epithelial cell membranes. In this research, the dipteran-specific Cry4Aa and Cry11A were shown, as expected, to be non-toxic to lepidopteran cells when activated with gut juices from *S. frugiperda*. However, these toxins acquired toxicity to lepidopteran cells after trypsin activation. These cell types appear, therefore, to express receptors capable of binding to the trypsin-activated Cry proteins used in this work. It is feasible that at least part of the specific toxic activity to dipteran insects is a consequence of the type of processing these toxins might have undergone in the insect gut. To confirm this hypothesis, binding assays should be carried out in future work. No toxicity of activated Cry4Aa and Cry11A was detected for a mammalian cell line. On the other hand, Cyt2Ba showed some toxicity to these cells, and in the presence of Cry4Aa and Cry11A, the toxicity was increased but was not statistically significant. Bti toxins are not expected to be harmful to humans, even if swallowed, because the toxin crystals need a pH of 10 or higher to be solubilized, while the human stomach has a pH of 1–3. Moreover, it is not plausible that the proteolytic pattern could activate a Bti toxin or that the protein would have a functional structure in a solution with such a low pH.

## Materials and Methods

### Bacteria and Eucaryotic Cells

The Brazilian *Bacillus thuringiensis* subsp. *israelensis* S-1989 and S-1806 strains were obtained from the *Bacillus* spp. bank of Embrapa Recursos Genéticos e Biotecnologia (Brasília, Brazil) as the source of *cyt2Ba*, *cry4Aa* and *cry11A* genes. Lepidopteran cells from *Spodoptera frugiperda*, IPLB-SF-21AE (primary explants of pupal tissue) [44], were obtained from Dr. Lois Miller, University of Georgia, US; *Lymantria dispar*, IPLB-LD-652Y (isolated from ovaries of the gypsy moth) [45] and *Bombyx mori*, BM-5 (isolated from ovaries of the silk worm) [46], were provided by Dr. Maria Elita de Castro, EMBRAPA-CENARGEN-Laboratório de virus de inseto, Brazil, The cells were maintained at 27°C in TC-100 medium supplemented with 10% bovine fetal serum (Gibco-BRL). *Aedes albopictus* cells C6/36 (a clone [47] derived from the Singh´s hatched minced larvae cell culture), obtained from Dr. Antônio Chaib, Laboratório Central de Saúde Pública (LACEN-DF), Brazil, were cultivated at 27°C in Leibowitz L15 medium, supplemented with 10% bovine fetal serum (Gibco-BRL). Human breast cancers cells MCF-7 [48], obtained from Laboratório de Morfologia, Universidade de Brasília, Brazil, were cultivated in DMEM (Sigma) medium supplemented with 10% bovine fetal serum at 37°C and 5% CO_2_.

### Construction of Expression Vectors for *Bacillus thuringiensis*

Plasmid DNA from Bti strains S-1989 and S-1806 were extracted by alkaline lysis [49]. The complete ORFs of *cyt2Ba* and *cry4Aa* genes were amplified by PCR using DNA from the S-1989 strain and specific oligonucleotide primers (cyt2BaHisBamHIForward-5′-GGATCC *ATG*CACCTTAATTTGAATAATTTT-3′; cyt2BaHisBamHIReverse-5′-GGATCCTT**AGTGGTGGTGGTGGTGGTG**ATACG ATTTTATTGGAT-3′;cry4AaForward-5′-CGGATCC *ATG*AATCCTTATCAAAAT AA-3′; cry4AaReverse-5′-CGGATCCTCACTCACTCGTTCATGAAATT-3′). In the same way, the complete ORF of the *cry11A* gene was obtained from the S-1806 strain using specific oligonucleotides (cry11AForward-5′-CAGGATCC *ATG*AATTATATGG AAGAT-3′; cry11AReverse-*5′-*CAGGATCCCTACTTTAGTAACGGATT-3′). *Bam*HI restriction sites were added to the oligonucleotide sequences (underlined text). The start codon of each gene is shown in italics (*ATG*) and the 6xHis tag codons fused to the *cyt2Ba* gene are shown in bold. To amplify the *cyt2Ba, cry4Aa* and *cry11a* genes, different PCR programs were performed using the respective three sets of oligonucleotides: ***cyt2Ba*** –94°C/5 min and 30 cycles of 94°C/1 min, 52°C/45 s, 72°C/1∶30 min and a final extension of 72°C/7 min; ***cry4Aa*** –94°C/5 min and 35 cycles of 94°C/1 min, 53°C/1 min, 72°C/2∶30 min and a final extension of 72°C/7 min; and ***cry11A*** –94°C/5 min and 30 cycles of 94°C/1 min, 53°C/1 min, 72°C/1∶30 min and a final extension of 72°C/7 min. Amplified fragments were cloned into the pGem-T®easy (Promega) vector, using *Escherichia coli* DH5-α® (Invitrogen) as a host, following the manufacturer’s instruction. DNA from recombinant plasmids was isolated [49] and sequenced (377-Applied Bio-system). The resulting genetically modified plasmids, pGemcyt2BaHis, pGemcry4Aa and pGemcry11A were digested with *Bam*HI, and then separated by electrophoresis in a 0.8% agarose gel. Fragments of approximately 800, 3,500 and 1,900 bp, corresponding to the *cyt2Ba*, *cry4Aa* and *cry11* genes, respectively, were purified using the GFX™ PCR DNA and Gel Band Purification Kit (GE Healthcare). The three genes were then separately cloned into the expression vector pSVP27A, kindly provided by Dr. David Ellar, University of Cambridge, UK [50], [51], and transformed into *E. coli* DH5-α®. The positive clones were selected by ampicillin resistance in culture medium (100µg/mL). The recombinant plasmids pSVP27Acyt2BaHis, pSVP27Acry4Aa and pSVP27Acry11A were isolated by alkaline lysis as described in [49]. The cloning of each gene was confirmed by restriction enzyme digestion followed by electrophoresis in agarose gels as described above.

### Expression, Purification and Solubilization of Cry and Cyt Proteins

An acrystalliferous Bti strain, 4Q7, kindly provided by Dr. Colin Berry, Cardiff University, UK, was used as a host for the constructed plasmids. The Bti cells were transformed with the recombinant plasmids pSVP27Acyt2BaHis, pSVP27Acry4Aa and pSVP27Acry11A by electroporation as previously described [52] with the following modifications. The electroporation parameters were adjusted on the BTX Electro Cell Manipulator™ 600 apparatus, using the following setup: 15 kV cm^−1^, 200 Ω e 25 µF. After electroporation, the cell suspensions were diluted in 1 mL LB broth and incubated with agitation (200 rpm) for 2 h at 28°C. After cell recovery by centrifugation, the pellets were resuspended and incubated on L-agar with 10 µg mL^−1^ chloramphenicol [48]. The positive clones were grown in selective NYSM media [53] with 10 µg/mL chloramphenicol at 30°C for 72 h. After this period, crystals and spores were separated in a discontinuous sucrose gradient according to protocol described below and as described elsewhere [12] with modifications. The bacterial cultures were collected and centrifuged at 16,000×*g* for 20 min and the supernatant was discarded. The pellets were resuspended and washed in 60 mL of a solution containing 0.3 M NaCl, 0.01 M EDTA pH 8.0 and centrifuged at 16,000×*g* for 20 min. This procedure was repeated twice; at the end of the third centrifugation the supernatant was discarded and the pellets were resuspended in 30 mL 1.0 mM PMSF. Fresh 1.0 mM PMSF solution was used to wash the samples by centrifugation at 16,000×*g* for 20 min. The sediments were then resuspended in TTN buffer (20 mM Tris HCl, 0.1% Triton X-100, 300 mM NaCl, pH 7.2). The samples were centrifuged at 25,000×*g* for 1 h in a sucrose gradient (84%, 79%, 72%, 67% and 54%). The protein bands corresponding to Cry11A, Cry4Aa and Cyt2BaHis, formed in the gradient, were collected and added to a 0.1% Triton X-100 solution. A new centrifugation at 25,000×*g* for 45 min was performed and the sediments were resuspended in 1,0 mM PMSF. The crystals of Cyt2BaHis and Cry11A were solubilized in 0.1 M Na_2_CO_3,_ pH 10.5 at 37°C for 1 h. The Cry4Aa crystals were solubilized in the same solution supplemented with the reducing agent 0.2% β-mercapto-ethanol. Any insoluble material was removed by centrifugation. The samples were neutralized with 0.1 M Tris-HCl pH 7.5 [54]. The 6xHis tag Cyt2Ba C-terminal fused protein was further purified by affinity chromatography using an agarose Ni-NTA column (The QIA expressionist™, QIAGEN), according to the manufactureŕs instruction, to remove any contaminants. The Bti S-1989 strain was also grown in the sporulation medium NYSM and the protein crystals were purified in a sucrose gradient, as described above for the individual Cry and Cyt proteins. The purified crystals were then solubilized with 0.2% β-mercapto-ethanol in 0.1 M Na_2_CO_3,_ pH 10.5 solution at 37°C for 1 h and then neutralized with 0.1 M Tris-HCl, pH 7.5. The samples were analysed by electrophoresis in a 12% SDS-PAGE (Mini-protean II – Biorad), following the manufacturer’s instruction.

### Toxin Activation

The samples containing the solubilized protoxins were quantified by fluorospectrophotometry using the NanoDrop 3300 apparatus together with the Quant-It™ Assay Kit (Invitrogen). The individually purified Cry toxins were activated by two methods. In the first method, the protoxins were incubated with pancreatic bovine trypsin (Sigma) at a 10∶1 ratio (w/w) for 2 h at 37°C. In the second activation method, the protease-containing gastric juice was obtained from ten *S. frugiperda* midguts following the procedure described in [55]. The Cry4Aa and Cry11A protoxins were incubated with the gastric juice at a 10∶1 ratio (w/w) for 2 h at 37°C. The samples obtained from both activation methods were dialyzed against distilled water using 0.025 µm membrane discs (Millipore™) and analyzed in a 12% SDS-PAGE. Purified Cyt2BaHis was also trypsin activated and dialyzed in the same conditions described for the Cry proteins. Furthermore, western blot analysis to check the Cyt2BaHis protein cleavage was carried out using a monoclonal anti-His antibody (GE Healthcare), following the manufacturer’s instruction. The solubilized wild type Bti protoxins were incubated with pancreatic bovine trypsin (Sigma) only at a 10∶1 (w/w) ratio for 2 h at 37°C, for protein activation, and dialyzed as above.

### Cytotoxicity Assays

The insect (IPLB-SF-21AE, IPLB-LD-652Y, BM-5, C6/36) and mammalian (MCF-7) cell lines, grown in 25 cm^2^ TPP flasks (Techno Plastic Products, Switzerland), were collected and added to 96-well plates (10^4^ cells/well). The culture medium of MCF-7 cells was removed and the cells washed with 1 mL PBS. A trypsin/EDTA (0.05%) solution was added to the cells, incubated at 37°C and 5% CO_2_ for 4 min and 1 mL of DMEM medium was added to stop trypsinization. The loose cells were centrifuged at 1,000×*g* for 3 min, resuspended in DMEM medium and added to 96-well plates (10^4^ cells/well). The activated Cyt2Ba, Cry4Aa and Cry11A toxins were added to the wells at predetermined concentrations. Cyt2Ba toxin was tested at two concentrations (5 or 20 µg/mL) separately or in combination with the other toxins. Cry4Aa and Cry11A toxins were used at the concentration of 20 µg/mL, individually or in the presence or absence of Cyt2Ba. The pool of wild type Bti activated toxins were incubated with all cell lines at the concentration of 5 µg/mL. All toxins were also incubated, at the mentioned concentrations, with different culture media in the absence of cells. Trypsin and gastric juice were individually incubated with C6/36 cells. All assays were carried out in triplicate. The time of all incubations with the three toxins as well as with the proteases, was 30 min. Furthermore, the culture media were incubated with CellTiter-Glo® Reagent from the CellTiter-Glo® Luminescent Cell Viability Assay kit (Promega) for 10 min to quantify the amount of ATP released to the media. The luminescence-based measurements were carried out in a Turner TD20/20 luminometer, with the following setup: delay time 5 s, integration time 20 s, sensitivity 50%.

### Mosquito Larvae

Neonate larvae of *A. aegypti* from the Rockfeller strain were provided by Embrapa Recursos Genéticos e Biotecnologia (Brasília, Brazil). The larvae were reared at room temperature (25°C) in autoclaved distilled water and fed on cat biscuit until they reached second instar.

### Bioassays

Sucrose-gradient isolated Cry11A and Cry4Aa crystals were added separately to 100 mL sterile tap water in disposable plastic cups containing 20 second-instar *A. aegypti* larvae, and mosquitocidal activities were determined after 24 h [56]. Serial dilutions of each crystal protein sample were used in the bioassays, and three replicates were performed for the seven doses tested, as well as for an untreated control group used as a negative control. The median lethal concentration for exposed populations was determined statistically by probit analysis using a program for PC (Polo Plus, LeOra Software). *A. aegypti* larvae were also exposed to a single dose of 20 µg/mL of each GJ-activated toxin (Cry11A and Cry4Aa), following the same method of incubation described above. All bioassays were performed in duplicate.

### Evaluation of Synergism

In order to identify potential synergistic effects, experimental LC_50_ (concentration of toxin responsible for 50% cell mortality) of each individual toxin and of the toxin mixtures (Cry4Aa/Cry11A, Cyt2Ba/Cry11A and Cyt2Ba/Cry4Aa) was estimated by probit analysis [57], using Polo Plus. Six doses ranging from 1 to 60 µg/mL of each toxin were incubated with insect cell lines following the method used for the cytotoxicity assays described above. For the Cry toxin mixture the ratio used was 1∶1, while for the Cry/Cyt mixtures the ratios were 0.8∶0.2. Three replicates were assayed with each dose. Synergistic interactions between the Cry toxins and between the Cry/Cyt were evaluated by the ratios of the theoretical LC_50_, obtained by Tabashnik’s equation [29], and the observed LC_50._ When the ratio was >1, the toxin interaction was considered to yield a synergistic effect as the toxicity was higher than the value predicted from individual additive toxicity. A ratio <1 meant that the interaction was antagonistic, whereas a ratio of 1 indicated only additive effects.
